The article "Research on a Health Care Personnel Training Model Based on Multilayered Knowledge Mapping for the Integration of Nursing Courses and Examinations" was retracted in 2023. Reasons: unreliable results or conclusions; concerns about the data; concerns about the peer review; concerns about the citations.

# Research on a Health Care Personnel Training Model Based on Multilayered Knowledge Mapping for the Integration of Nursing Courses and Examinations

**DOI:** 10.1155/2022/3826413

**Published:** 2022-02-09

**Authors:** Qingna Lv, Yanyun Zhang, Yanyan Li, Yang Yu

**Affiliations:** ^1^Nursing Department, The Second Affiliated Hospital of Dalian Medical University, Dalian, Liaoning 116023, China; ^2^College of Nursing, Inner Mongolia Minzu University, Tongliao 028000, Inner Mongolia Autonomous Region, China; ^3^College of Nursing, Chongqing Medical and Pharmaceutical College, Shapingba, Chongqing 401331, China

## Abstract

While nursing courses provide a convenient and quick way to learn, they can also be overloaded with resources that can cause learners to become cognitively disoriented or have difficulty choosing nursing course. This paper proposes to fully explore learners' interests in the case of sparse data by fusing knowledge graph technology and deep recommendation models and adopt knowledge graph to model nursing courses at the semantic level so as to correspond the set of nursing courses to the knowledge graph and solve the problem of lack of logical knowledge relationships. Due to the specificity of its positions, the nursing profession must accurately position the nursing professional curriculum standards in the process of determining the talent cultivation model based on the nursing professional positions and the admission requirements for nursing practice qualification. Through linear feature mining based on the knowledge graph, entities and relationships are used to intuitively display the interest paths of nursing professional learners and enhance the interpretability of recommendations.

## 1. Introduction

Vocational education is the foundation of human resource construction. Vocational nursing education is vigorously developed to train high-quality skilled and practical nursing personnel for society in order to meet the growing health and hygiene needs of the people. Because of the special nature of its service targets (patients), nursing vocational education requires practitioners to have national nurse practice qualifications. Therefore, we should reform and innovate the training mode of nursing talents, take employment as the orientation, take competence as the basis, take theoretical knowledge and practical skills competition as the grasp, integrate the dual requirements of nursing positions and nursing practice qualification examination into the teaching system of nursing professional courses [1], promote students' interest in professional theory learning, and focus on improving students' vocational skills through theoretical knowledge and practical skills competition, which is conducive to improving graduates' employ ability [2]. In other words, the theory is guided by the operation, and the theory is constantly verified and enriched in the operation, so as to achieve the teaching effect of “circular teaching, learning, and doing in one” [3], which is the integration of theory and practice.

The article "Research on a Health Care Personnel Training Model Based on Multilayered Knowledge Mapping for the Integration of Nursing Courses and Examinations" was retracted in 2023. Reasons: unreliable results or conclusions; concerns about the data; concerns about the peer review; concerns about the citations.

All nursing students who have completed the course and are currently enrolled in the course are required to take part in the theoretical knowledge competition of the subject. The competition is divided into two stages, the preliminaries and the final, and the results are linked to class and individual merit. Through the competition, students can consolidate their professional knowledge, improve their ability to learn independently, and enrich the second classroom; at the same time, it also allows students to experience the atmosphere of the nursing examination in advance and achieve the effect of simulating the nursing examination [4]. In addition, by participating in the preliminaries collectively, it not only stimulates the class' sense of collective honour and improves the cohesion of the class, but also creates a good learning atmosphere within and between classes, which greatly enhances students' interest in professional learning and improves the quality of teaching in general [5].

Include professional skills assessment and competition in regular teaching sessions so that school skills competitions can be dovetailed with provincial and national skills competitions and focus on improving the teaching level of students' vocational skills: nursing is a highly practical profession, and practical teaching sessions are a key part of training nursing students to become qualified clinical nurses. Through skill competition activities, the teaching level of teachers and the clinical practice ability of students can be improved [6].

Develop a practical competition plan to ensure that the skills competition is put into practice:

Take the training of young teachers as a breakthrough to build a “two-teacher” teaching team: (1) focus on the training of young teachers' nursing skills. The training of young teachers' nursing skills is incorporated into the school-based training plan for young teachers, and a combination of one-to-one personal coaching and group training is adopted to train young teachers in nursing skills so as to ensure “double-teacher” teaching and improve the quality of teaching in practical classes [7]. (2) Regularly assess the basic nursing skills of young teachers who have graduated from the nursing program. Every semester, we routinely conduct basic nursing skills assessment for young teachers graduating from nursing majors so as to help young teachers master all basic nursing skills as soon as possible. (3) Gradually cultivate a nursing faculty team that combines teaching the ability to excel in pretournament coaching. On the basis of completing daily teaching work, senior and experienced teachers are organised to conduct in-depth research on the training mechanism of the nursing skills competition so as to cultivate a nursing teacher team that integrates teaching with the ability to provide pretournament guidance, making it a “strong guard and capable of winning in times of war” that is able to teach well in normal times and put in timely efforts to provide guidance to students in pretournament training. (4) Conduct nursing skills competition for young teachers. On the basis of the regular teaching competitions and lecture competitions for young teachers in nursing course, the nursing skills competitions for young teachers have been arranged in a planned manner to effectively promote the healthy growth of a skilled teaching team [8].

The article "Research on a Health Care Personnel Training Model Based on Multilayered Knowledge Mapping for the Integration of Nursing Courses and Examinations" was retracted in 2023. Reasons: unreliable results or conclusions; concerns about the data; concerns about the peer review; concerns about the citations.

Scientifically formulate practical training plans to promote a good match between skills competitions and practical training teaching: (1) Highlight the teaching of the nursing professional course “Fundamentals of Nursing.” When formulating and implementing the teaching plan, the number of hours should be increased appropriately; in terms of teacher deployment, a new and old partner is adopted so that young teachers can learn while doing under the premise of simulating the teaching of the old teachers throughout the course. (2) Adhere to the combination of classroom operation and after-class practice. Because of the limited time for classroom practice, in order to ensure that students master each nursing skill in time, on the basis of classroom demonstration and practice, a large number of extracurricular practice exercises are reasonably arranged for students, and “those who are able are teachers” and mutual help and learning are strongly advocated among students [9]. (3) Include nursing skills assessment in the assessment of nursing courses. In order to stimulate students' enthusiasm for nursing practice, the nursing skills' assessment is included in the evaluation mechanism and accounts for 50% of the total grade of the course. (4) Routine nursing skills competitions are held throughout the department. In the first semester of each academic year, the nursing skills competition of the whole department is carried out routinely, not only to test the results of nursing skills training and stimulate teachers' enthusiasm for teaching and students' motivation for learning, but also to select participants or reserves for the school to participate in the provincial or even national nursing skills competition in the first half of the following year [10].

The article "Research on a Health Care Personnel Training Model Based on Multilayered Knowledge Mapping for the Integration of Nursing Courses and Examinations" was retracted in 2023. Reasons: unreliable results or conclusions; concerns about the data; concerns about the peer review; concerns about the citations.

This study constructs a knowledge graph of nursing professional courses through the nursing professional course dataset, uses the knowledge graph information to carve the semantic network relationship of the nursing professional course recommendation domain, and proposes a set of knowledge graph-enhanced nursing professional course recommendation methods. The aim is to ensure the accuracy of the recommendations while recommending personalised and knowledge-logical nursing courses for learners. The method has certain theoretical and practical implications.

In terms of theory: (1) Innovative application of knowledge mapping technology: based on the characteristics of nursing courses which are logically related and hierarchical, this paper applies knowledge mapping technology to nursing course recommendations, making full use of the triadic relationship of the mapping to mine learners' preferences and learning paths [11]. For example, Java is a high-level programming language with object-oriented properties, and Python is included in the set of high-level object-oriented programming languages. We can find learners' nursing course preference paths by mapping nursing course to knowledge graphs [12].

## 2. Related Work

The development of nursing education has made up for the shortcomings of traditional education, but with the advent of the era of big data, nursing education platforms have gradually emerged with problems such as the uneven quality of nursing courses and the difficulty of choosing from a large number of them. Reference [13] argues that a nursing course recommendation system is a necessary tool in the student learning process, as a guide for students to choose from. In the era of personalised education, scholars are increasingly interested in recommending nursing courses and resources in the field of teaching and learning. From the perspective of recommendation, it can be divided into nursing course recommendation based on learners' interests and nursing course recommendation based on knowledge paths. In [14], a personalised learning resource recommendation tool was developed by constructing a learner model in a digital learning environment based on an e-book package. Reference [15] is based on the simulated data of the MOOC platform and the customized expertise mapping. We discussed and analyzed how to combine learners' historical learning data and expertise mapping information in the MOOC to generate the best learning path recommendations. Reference [14] proposed learner profile modelling based on interest mapping to build a personalised recommendation system for nursing course in a cold environment. In [16], a comprehensive comparative analysis of commonly used recommendation techniques and algorithms in the field of educational technology is presented, and optimization suggestions are made according to the current problems in the field of nursing course recommendation. At the same time, various deep learning methods and neural network models were also applied to the field of nursing course recommendation. In [17], CNN networks were used to extract user-relevant implicit factors from text, and the split Bregman iterative method was introduced to optimise the model, which was eventually able to achieve automatic recommendation of learning resources. Reference [18] improved the recommendation results of mooting by adding the information features of learners into the Neum model and proposed using convolutional neural networks to predict students' learning performance. In [19], considering the time-series nature of learners' course selection records, an LSTM network was used to extract learners' learning characteristics from time-tagged learners' historical course selection data and then predict the nursing course that learners might choose. The LSTM network was used to extract learners' learning characteristics from learners' historical course selection data with temporal labels and then to predict which nursing course learners might choose [20]. Reference [21] takes junior high school physics as an example. We combined students' learning styles and proficiency tests to achieve nursing course resource recommendations based on the knowledge structure of physics subjects. The knowledge embedded in the MOOC resources was constructed into a knowledge graph, and then the MOOC resources were bound to the entities on the knowledge graph to achieve a customized learning path by combining the learning objectives of the learners [22].

The article "Research on a Health Care Personnel Training Model Based on Multilayered Knowledge Mapping for the Integration of Nursing Courses and Examinations" was retracted in 2023. Reasons: unreliable results or conclusions; concerns about the data; concerns about the peer review; concerns about the citations.

## 3. Knowledge Graph Construction Techniques

Knowledge graph-related technologies can be divided into five subdomains: knowledge representation and modelling, knowledge acquisition, knowledge fusion, knowledge graph query reasoning, and knowledge graph application, whose basic technology system is shown in Figure 1.

As this study requires the construction of a recommended knowledge graph for nursing courses, the main introduction to the techniques involved in the construction of the knowledge graph will be given.

The construction of knowledge graphs is divided into top-down and bottom-up approaches: top-down extracts high-quality triadic information from texts such as encyclopaedias, while bottom-up extracts data information that meets the requirements from existing graph databases. In terms of the construction process, there are three main stages: knowledge extraction, knowledge fusion, and knowledge processing.

### 3.1. A Preliminary Knowledge Mapping of the Nursing Curriculum

The main data source for building the knowledge map of nursing courses is the classical knowledge map DBpedia, which is an English knowledge map, and the seed set of the map we obtained is a collection of mixed Chinese and English subscripts, so direct translation and alignment may result in some subscripts not corresponding to entities due to inaccurate translation. In order to improve the accuracy of entity alignment, we use the following approach to entity alignment.

Using seeds of aligned successful entities, we searched the DBpedia knowledge graph for entities in the disambiguation dataset and their one-to-five level neighbours (tail entities in a triad) and then extracted all triad information related to these entities. To reduce irrelevant data in the knowledge graph, we filtered the crawled triad information from a relational perspective [23]. The main process is as follows: firstly, the technical class entities are selected from the entity seed and all the trial information with them as the head entities are crawled using the technical class entities. Then, the relationships in the triad information are counted and ranked in terms of frequency, and the top 34 relationships with the highest frequency ranking are selected as the set of standard relationships. Finally, 34 standard relations are used to filter the remaining triples; that is, only the triples related to the standard relations are retained. Finally, the filtered data were collated to form the initial version of the knowledge map of the nursing curriculum as shown in Figure 2.

## 4. Nursing Course Knowledge Mapping Supplement

In order to ensure the quality of the complementary mapping information, there are three basic conditions for this complementary work. (1) Quantitative limitation: the triad formed by the new entities must have more than two and less than six triads of information. Too much or too little information about the entity triad is not conducive to the construction of the map. (2) Entity qualification: the tail entity in the complemented triad must be an entity in the seed entity set. (3) Relationship domain qualification: the types of relationships in the complemented triples are restricted to the original relationship domain. Firstly, we obtain the Baidu encyclopaedic descriptions of all the subterms from the Baidu encyclopaedia. The set of tail entities associated with the subterms is extracted from the encyclopaedia descriptions. In order to ensure the integration and interaction with the initial knowledge graph, only the entities in the seed entities were selected as the tail entities in the triad information, and the remaining information was eliminated. Secondly, in order to ensure that the manually completed information is consistent with the structure level of the original nursing curriculum knowledge map, the 34 relationships are classified into the following categories according to their nature, and the completed relationships are assigned values based on the set of relationships. The specific categories are shown in Table 1.

The article "Research on a Health Care Personnel Training Model Based on Multilayered Knowledge Mapping for the Integration of Nursing Courses and Examinations" was retracted in 2023. Reasons: unreliable results or conclusions; concerns about the data; concerns about the peer review; concerns about the citations.

## 5. Knowledge Graphs for Fusing Networks of Co-Reactors

The core idea of the RippleNet algorithm is to find the user's interest by using the multilayer relationships of the seed entities diffused in the knowledge graph. Features. The RippleNet algorithm is based on the idea of using the multilayered relationships of seed entities to find features of interest to the user in the knowledge graph. In particular, related entities in the overlapping part of the hierarchy resulting from the “ripples” of the seed produce a phenomenon similar to “interference enhancement” in physics [24].

In the case of nursing course names and news headlines, which do not correspond to specific entities per se but do correspond to sets of entities in pairs, we found a specific co-occurrence of entities. The presence of the name of the nursing course is particularly evident in the series of nursing courses “Android Must Learn AsyncTask Base Validation,” “Androiddroid-Reacquaintance Activity,” where the set of selected courses corresponding to the entity “Android” was hit several times directly and even played a more decisive role in the process as shown in Figure 3.

The RippleNet algorithm only takes into account the implicit interest that can be portrayed by the seed set of entities and their multilayered neighbours, ignoring the explicit interest that users already show in the selection of nursing course names. Therefore, to address the specific “one-to-many” nature of the “set of nursing course name entities,” we introduce a coreality network, the co-net, based on the RippleNet algorithm, to retrospectively capture the explicit interests of users. We propose a fusion of coreality entities and co-net to capture the explicit interests of users. We therefore propose a knowledge graph recommendation model, Ripple mlp+, that incorporates the coreality network. Ripple mlp+ is based on the Ripple_m model and optimises the knowledge graph learning module by introducing the coreality network co-net to populate the original knowledge graph. The optimized network is shown in Figure 4.

The article "Research on a Health Care Personnel Training Model Based on Multilayered Knowledge Mapping for the Integration of Nursing Courses and Examinations" was retracted in 2023. Reasons: unreliable results or conclusions; concerns about the data; concerns about the peer review; concerns about the citations.

The shaded part of the figure is the real body network co-net, which contains the nursing course entities as well as the nursing course subword entities. For the training of the coreality network and the determination of the edge weight, we use the same approach as for the training of the knowledge graph. The co-occurrence network information is analogous to the knowledge graph triad, and the relationships are assigned as “technical clauses” and “non-technical clauses,” thus forming (nursing course name, technical clause, technical entity) and (nursing course name, non-technical clause, non-technical entity). The set of triples is called *Co*_*l*_^1^.

The weight of the relationship from the nursing course name to the nursing course subword can be calculated by the following formula:

(1) $$\begin{array}{c} P_{i}=\text{soft }\max\left(C_{R}^{T}R_{i}h_{i}\right)=\frac{\exp\left(C_{R}^{T}R_{i}h_{l}\right)}{\sum_{\left(h,r,e\right)\text{Î}C_{0}^{1}}\exp\left(C_{R}^{T}Rh\right)}. \end{array}$$

Characteristics of learners' interests on coreality body networks *O*_*l*_^1^ are expressed as

(2) $$\begin{array}{c} o_{l}^{0}=\sum_{\left(C,r,e\right)\text{Î}Co_{l}^{1}}P_{i}e_{i}. \end{array}$$

Learner profile *L*_*R*_ is expressed as

(3) $$\begin{array}{c} L_{R}=O_{l}^{0}+\overset{H}{\underset{k=1}{\sum }}O_{l}^{k}\\ =\overset{H}{\underset{k=0}{\sum }}O_{l}^{k}. \end{array}$$

The goal of the recommendation algorithm is to predict the potential interest of learner *I* in a nursing course *c* that he has not chosen before. This means that the model is trained to produce a prediction function ${\hat{y}}_{lc}=F\left(1,c|\Theta ,Y,G,Co\right)$, where ${\hat{y}}_{lc}$ denotes the probability of interaction between learner *l* and nursing course *c* as predicted by the model, and ⊙ denotes the parameters of the function *F*.

## 6. Model Optimisation

In order to train and optimise the model, we obtain equation (4) based on the maximum posterior probability estimate. In order to obtain an optimal solution for the model, the posterior probability is maximised. That is, let equation (3) have a maximum value.

(4) $$\begin{array}{c} \max p\left(\Theta |Y,G,Co\right). \end{array}$$

An expansion of equation (4) from the Bayesian formula gives

(5) $$\begin{array}{c} \max p\left(\Theta |Y,G,Co\right)=\frac{p\left(\Theta ,Y,G,Co\right)}{p\left(Y,G,C_{0}\right)}\propto p\left(\Theta \right)\cdot p\left(G,Co\Theta |\right)\cdot p\left(Y\Theta |,G,Co\right). \end{array}$$

The second term *p*(*G*, *Co|*Θ) is the probability of obtaining the knowledge graph *G* and the corealistic body network **Co** if 0 is known.

(6) $$\begin{array}{c} p\left(G,Co|\Theta \right)=\prod_{\left(h,r,t\right)\in G\cup c_{0}}p\left(\left(h,r,t\right)\Theta \right)\\ =\prod_{\left(h,r,t\right)\in G\cup C_{0}}N\left(I_{\left(h,r,t\right)}-h^{T}RT,\lambda_{2}^{-1}\right), \end{array}$$

where *I*(*h*, *r*, *t*) is an indicator function. The value is 1 when the triad (*h*, *r*, *t*) is a true triad (i.e., when the triad belongs to a knowledge graph collection or a coreality network) and 0 when the triad (*h*, *r*, *t*) is a false triad, and we expect *I*_(*h*, *r*, *t*)_ − **h**^**T**^**RT** to be as close to 0 as possible in order to better reproduce the information of the graph and coreality network.

The article "Research on a Health Care Personnel Training Model Based on Multilayered Knowledge Mapping for the Integration of Nursing Courses and Examinations" was retracted in 2023. Reasons: unreliable results or conclusions; concerns about the data; concerns about the peer review; concerns about the citations.

The third term *p*(**Y***|*Θ, **G**, **Co**) is a dichotomous similar likelihood function, in order to evaluate the effect of the model on the classification (course selection or not).

## 7. Experimental Results and Analysis

### 7.1. Comparison with Their Methods

In order to verify the effectiveness of the algorithm proposed in this study, we chose other algorithms as the experimental benchmark method for experimental comparison with the algorithm proposed in this paper. The higher AUC and ACC values of the experimental results represent the better performance of the model, and the experimental results are shown in Table 2. The results show that the performance of both Ripple_mlp+ and Ripplejmlp is higher than that of the benchmark algorithm [25].

For the NCF model, the Ripple_mlp model optimises the generalised matrix decomposition in the NCF model into a knowledge graph-based feature extraction, and the new model incorporates more knowledge graph information to improve the accuracy of the recommendation results. Similarly, the results of the NMF, a two-network model with “serial” processing, also failed to outperform the Ripple mlp model. This phenomenon also supports the idea that providing more diverse information to the recommendation system helps the model to obtain descriptive data, build more accurate feature models, and ultimately obtain better recommendation results.

The two models proposed in this study, Ripple map and Ripple mlp+, obtain the optimal AUC quickly using only one epoch, which also shows that the models are able to capture user interest features from a small amount of data very quickly and have a significant advantage over other benchmark methods in terms of model convergence time [26].

### 7.2. Performance Analysis

In addition to the comparison with the benchmark method, we also explored the effect of parameter settings on model performance by adjusting the parameter values associated with the Ripple_mlp + model.

(1) The feature dimensions of depth perceptron and the different settings of neurons have an impact on the performance of the model. We varied the feature dimension dim from 8 to 32, keeping the other parameters fixed, and were able to find that the best AUC values were achieved when *d* = 16. Either too long or too short a feature dimension will reduce the performance of the model.

The article "Research on a Health Care Personnel Training Model Based on Multilayered Knowledge Mapping for the Integration of Nursing Courses and Examinations" was retracted in 2023. Reasons: unreliable results or conclusions; concerns about the data; concerns about the peer review; concerns about the citations.

The number of neurons in each layer was halved layer by layer to investigate the effect of the number of neurons on the experimental results. It was found that the best results were obtained when the number of neurons of the deep perceptron was set to [12864,32,16], regardless of the value of the feature dimension dim. This also shows that there is an upper limit to the learning and fitting ability of the deep perceptron for the nonlinear interaction function, and the use of appropriate network parameter settings can prevent the deep perceptron from underlearning or overfitting, and the variation of the settings is shown in Figure 5.

In modelling the learner interest profile, we obtained a vector representation of learner interest by summing up each level of interest at a distance *k* from the learner's chosen nursing course. As the distance *k* increased, more and more triadic information was incorporated into the learner interest representation. Each layer of triads on the water wave brings a wealth of information about the representation of learner interest features. However, when the value of *k* exceeds a certain value, too much noise data is introduced, and the impact of noisy data on the model performance may outweigh the enhancement of the model by the valid information.  Table 3 shows how the AUC of the model changes as the number of water wave layers *k* varies. (*k* = 0) represents the coreality body network layer. Analysis of the data in Table 3 shows that when the value of *k* is too small, there will be insufficient training of model learning; when the value of *k* is too large, it will bring invalid data to affect the experimental results. Therefore, when training the characteristics of the knowledge graph, the model should be trained with an appropriate *k* value (optimal for *k* = 2 for this model).

### 7.3. Experimental Data Impact

The quality of the dataset will have a great impact on the experimental results of the model as it is the basis for model learning. In order to investigate the model's ability to perform on datasets with different sparsity levels, we obtained four datasets with different sparsity levels using different proportional sampling methods on the cleaned datasets. The total number of learners in the sample was kept at 5000 and the number of nursing course was 937. Four datasets after sampling are shown in Table 4.

The article "Research on a Health Care Personnel Training Model Based on Multilayered Knowledge Mapping for the Integration of Nursing Courses and Examinations" was retracted in 2023. Reasons: unreliable results or conclusions; concerns about the data; concerns about the peer review; concerns about the citations.

Based on different sparse datasets, we experimented three times using the Ripple_map + model and took the average of the three experimental results for comparison. The experimental results are shown in Figure 6.

The Ripple_mlp + model achieves an AUC of over 88% and an accuracy of over 80% for both sparse and dense datasets, making its overall performance relatively stable [27]. However, the sparsity of the dataset still affects the performance of the model. As the sparsity of the dataset decreases, it means that the interaction data in the dataset brings more effective information, so the indicators of the model show an increasing trend; however, as the data gradually becomes denser, the evaluation indicators of the model decrease. We believe that there are two reasons for this phenomenon: (1) The increase of data does not mean the increase of valid information from the dataset itself. On the contrary, the increase in data may also bring a lot of noise data. Therefore, excessively dense data set may lead to a decrease in model metrics. (2) The relevant parameters within the model are considered.

The distribution of nursing students' course learning effects is shown in Figure 7. By conducting research on the content of nursing course related to the nursing examination syllabus and nursing examination questions, it is conducive to linking the teaching of nursing courses with the examination syllabus. This will help to link the teaching of nursing courses with the examination syllabus and improve the quality of teaching of nursing course.

Analysis of the revised and new diseases in the nursing examination syllabus is conducive to teachers' teaching in different disciplines: By investigating and studying the new and revised diseases in the new syllabus and the changes in the disciplines to which they belong, it is conducive to teachers' teaching in different disciplines, grasping the new priorities and adding new contents so as to achieve the purpose of integrated teaching reform in the study of the syllabus and teaching [28]. A study is carried out on the correlation between the nursing examination and the nursing practice teaching reform to promote the organic integration of clinical practice and school teaching: Based on the nursing examination syllabus and the needs of nursing positions, the classification of nursing vocabulary is shown in Figure 8.

Our research meets the requirements of the nursing examination outline. The research of this paper is conducive to the implementation of the nursing curriculum of target teaching. For example, the nursing curriculum based on the combination of engineering and practical training can improve the application and development of the nursing examination outline and teaching materials. The textbooks for the “combined engineering” professional courses in nursing and their corresponding experimental and practical training are developed on the basis of the syllabus of the nursing examination and the results of the relevant teaching reform.

The article "Research on a Health Care Personnel Training Model Based on Multilayered Knowledge Mapping for the Integration of Nursing Courses and Examinations" was retracted in 2023. Reasons: unreliable results or conclusions; concerns about the data; concerns about the peer review; concerns about the citations.

## 8. Conclusions

This paper proposes to fully explore learners' interests in the case of sparse data by fusing knowledge graph technology and deep recommendation models and adopt knowledge graph to model nursing courses at the semantic level, so as to correspond the collection of nursing courses to the knowledge graph and solve the problem of lack of logical knowledge relationships. In the process of determining the talent cultivation model, the nursing profession, due to the special nature of its positions, must accurately position the nursing professional curriculum standards according to the nursing professional positions and the requirements for admission to nursing practice qualification.

## Figures and Tables

**Figure 1:** Knowledge graph technology system.

**Figure 2:** Flowchart of Wikipedia-assisted alignment.

**Figure 3:** Network diagram of nursing course subword entities.

**Figure 4:** Combined knowledge graph and coreality body network graph G + Co.

**Figure 5:** Variation of model AUC with the value of (d) num_factor setting.

**Figure 6:** Effect of datasets with different sparsity on model's performance.

**Figure 7:** Distribution of nursing students' course learning outcomes.

**Figure 8:** Classification of professional nursing vocabulary.

**Table 1:** Table of knowledge graph relationship categories.

Relationship type	Relational meaning	Triples example
Inclusion relation	Relationship between whole and part	Baseadapter, category android adapter
Belonging relationship	Relationship between part and whole	Android adapter, category zh, baseadapter
Application relationship	Relationship between technology and application	CSS technology, usage, website development
Development relationship	Relationship between technology and developers	Baidu map, developer, Baidu
Reference relation	Relationships other than the above relationships	Impress. js, Language JavaScript

**Table 2:** Comparison table of experimental results with the benchmark algorithm.

Model	AUC	ACC	Best_epoch
NCF	0.8817 (−0.37%)	0.8017 (−0.32%)	2.4
RippleNet	0.8822 (−0.32%)	0.8012 (−0.39%)	7.8
NFM	0.8444 (−4.1%)	0.7689 (−3.62%)	144.1
Ripple_mlp	0.8854	0.8051	1
Ripple_mlp+	0.8907 (+0.53%)	0.8110 (+0.59%)	1

**Table 3:** Effect of the number of water wave layers *k* on the experimental results.

*k* value	0	1	2	3
Model AUC	0.8638	0.8644	0.8651	0.8645

The article "Research on a Health Care Personnel Training Model Based on Multilayered Knowledge Mapping for the Integration of Nursing Courses and Examinations" was retracted in 2023. Reasons: unreliable results or conclusions; concerns about the data; concerns about the peer review; concerns about the citations.

**Table 4:** Four datasets sampled with different levels of sparsity.

Data set	Total interactions	Average number of interactions	Sparsity (%)
Sparse data set	163527	32	96.51
Sparse dataset	209494	41	95.53
Dense data set	286025	57	93.89
Dense data set	521750	104	88.86

## Data Availability

The authors did not obtain analytical permission from the data provider because of trade confidentiality.
